The article "Isokinetic Assessment of Shoulder Joint Strength Ratios in Male Recreational Weightlifters: A Cross-Sectional Study" was published in 2022. Journal: Appl Bionics Biomech.

# Isokinetic Assessment of Shoulder Joint Strength Ratios in Male Recreational Weightlifters: A Cross-Sectional Study

**DOI:** 10.1155/2022/6106943

**Published:** 2022-06-13

**Authors:** Osama R. Abdelraouf, Marwa Y. Ebrahim, Amr A. Abdel-aziem, Soheir M. Abdel-Rahman, Ahmed S. Yamani, Ahmad A. El Askary

**Affiliations:** ^1^Physical Therapy program, Batterjee Medical College, Jeddah 21442, Saudi Arabia; ^2^Department of Biomechanics, Faculty of Physical Therapy, Cairo University, Giza 12613, Egypt; ^3^Department of Physical Therapy, College of Applied Medical Sciences, Taif University, P.O. Box 11099, Taif 21944, Saudi Arabia; ^4^Department of Clinical Laboratory Sciences, College of Applied Medical Sciences, Taif University, P.O. Box 11099, Taif 21944, Saudi Arabia

## Abstract

**Background:**

Isokinetic strength imbalance is a risk factor for movement dysfunctions and injuries related to shoulder complex. The effects of recreational weightlifting on developing the imbalances between the shoulder muscles are not yet known.

**Objectives:**

To investigate the isokinetic concentric shoulder muscle strength values (peak torque normalized to body weight) in recreational weightlifters (RWL) and to compare the shoulder muscles agonist/antagonist ratios with nonweightlifters.

**Methods:**

Thirty male RWL with mean age, weight, height, and body mass index (BMI) of 21.56 years, 84.25 kg, 175.34 cm, and 26.51 kg/m^2^, respectively, matched with nonweightlifters served as a control group. The normalized concentric peak torque values of shoulder flexors, extensors, abductors, adductors, and internal and external rotators were measured at angular velocity 120°/sec by using Biodex isokinetic system. Moreover, the agonist/antagonist strength ratio for all muscle groups were calculated.

**Results:**

The normalized peak torques of RWL group were significantly greater than the control group (*p* < 0.05). The abductor/adductor and external rotator/internal rotator ratios of the RWL were significantly lower than the control group (*p* = 0.008 and 0.009, respectively). Conversely, there was no significant difference between both groups in relation to the flexor/extensor ratio (*p* = 0.259).

**Conclusion:**

These results suggested that the recreational weightlifting exercises place trainees at risk of muscle imbalances. Therefore, the restoration of a normal concentric abductor/adductor and external rotator/internal rotator strength ratios may decrease the risk of possible shoulder injury.

## 1. Introduction

Weightlifting is widely used for various health benefits such as sports [1], injury rehabilitation, maintenance of cardiorespiratory and muscular fitness [2], and the development of muscle hypertrophy and shaping [3]. It is estimated that almost 45 million Americans are regularly engaged in weight training programs [4]. However, weightlifting is associated with numerous injuries. The lower back followed by the shoulder and knee joints are the most frequently affected areas [5]. According to Kerr et al. [6], shoulder injuries account for 36% of all injuries and disorders in the weightlifting trainees.

The article "Isokinetic Assessment of Shoulder Joint Strength Ratios in Male Recreational Weightlifters: A Cross-Sectional Study" was published in 2022. Journal: Appl Bionics Biomech.

Two main types of exercises are incorporated in weightlifting training programs: complementary exercises that have movement patterns similar to the competitive lifts (e.g., hang/power snatch) and supplementary exercises (e.g., overhead presses) that target synergistic muscle groups [7]. Many muscle contractions are performed by the same major muscle groups during each training session. The frequency of lifting might exceed evidence-based recommendations for improving muscular strength and power [2]. Most adopted weightlifting training programs are designed based on multiple sets of submaximal to maximal muscle loading to match the demand during competitive practices. It was estimated that weightlifters performed between 1400 and 4000 maximal attempts, and 450 and 460 failed supramaximal attempts each year of training [8].

Muscular balance is crucial for normal shoulder function. Both static and dynamic situations of the shoulder joint depend, to a great extent, on balanced muscular strength and power. Dynamic situation is a function of deltoid muscle as prime mover balanced by the force of gravity and infraspinatus, subscapularis, and teres minor muscles [9]. In the same context, the balance between trapezius and serratus anterior muscles serves as the primary mechanism in upward rotation of scapulothoracic joint, which is necessary for arm elevation [10]. Disturbance of the previously mentioned force couples is a common risk factor in many shoulder injuries [11, 12]. In recreational weight training (RWT), muscle imbalance results from training large muscles called mirror muscles (pectoralis, deltoid, and upper trapezius muscles) at the expense of the shoulder complex stabilizers [13]. This imbalance exposes the recreational weightlifting trainees to a high risk of injuries [14].

Muscular imbalance and improper technique can both impair athletes' performance and put them in danger. A prolonged clean and jerk motion, which is thought to be the fundamental movement for weightlifting, appears to aggravate muscular imbalances, leading to an increased risk of injury [15]. A recent study reported imbalance of the isokinetic profiles of rotator cuff muscle strength and power between both upper limbs in adolescent weightlifters [16]. Muscle strains, ligament sprains, pectoralis major tendon ruptures, distal biceps tendon ruptures, chronic shoulder pain, and capsulolabral injuries are all common upper extremity injuries in resistance training athletes. While each injury is unique in its anatomic location and mechanism, they are all preventable with proper exercise technique, safety, and muscle balance maintenance [4].

The article "Isokinetic Assessment of Shoulder Joint Strength Ratios in Male Recreational Weightlifters: A Cross-Sectional Study" was published in 2022. Journal: Appl Bionics Biomech.

A literature review showed that no previous studies have investigated muscle imbalances in RWL. Moreover, this may help physical therapists, strength coaches, and athletic trainers in designing an effective and safe shoulder resistance training. So, the aim of the current study was to assess the isokinetic concentric shoulder muscle-normalized torque values and to compare the agonist/antagonist ratios of RWL with nonweightlifters. It was hypothesized that there will be a difference between groups in terms of normalized isokinetic torques in the favor of RWL group with no difference in terms of the agonist/antagonist ratios.

## 2. Methods

### 2.1. Participants

This cross-sectional study was conducted on thirty male RWL with age range from 18 to 30 years (study group) who were recruited from local fitness centers. They were matched with a similar number of nonweightlifter (healthy) subjects with similar demographic data as the control group. The weightlifters should be involved in upper extremity resistance weight training at least three times per week for the previous six months [17]. Participants were excluded if they used anabolic steroids and participated in professional bodybuilding, competitive power lifting, or other overhead sports. The nonweightlifters were excluded if they participated in a formal type of upper extremity resistance training exercise and if they had a history of upper extremity or neck symptoms. Shoulder pain or injury at the time of the study was an exclusion criterion for both groups. Demographic data of the study and control groups are shown in Table 1.

Before the beginning of the study, the local university's ethical committee reviewed and approved all procedures (ID:P.T.REC/012/00728). Participants were oriented about the purpose and procedures of the study and signed an informed consent. Using G∗Power 3.1 software, the sample size was calculated to be 30 participants in each group. The alpha value, power, and effect size were set at 0.05, 0.90, and 0.85, respectively.

### 2.2. Procedures

For data collection, the nondominant arm was used to avoid the effect of dominance on isokinetic strength [18]. Based on motor skills, dominant arm was defined as the one preferred for daily activities such as eating, writing, cutting, and catching [19]. The shoulder exercises and the number of exercise repetitions each participant performs in his routine workout were provided. Different types of upper extremity weight training exercises (lever inclined chest press, butterfly, bench press with barbell, dumbbell one arm row, cable standing fly, bench press with dumbbell, decline and incline bench press with barbell or with dumbbell, dumbbell fly, lever shoulder press, assisted pull up, reverse butterfly, neck press with dumbbell, lateral deltoid raise, reverse fly with dumbbell, diagonal lateral cable raise, upright cable row, and cable external rotation) were presented in special sheet from which participant chose exercises he usually practiced in his weight training. A summary of the study procedures is presented as a flowchart (Figure 1).

The article "Isokinetic Assessment of Shoulder Joint Strength Ratios in Male Recreational Weightlifters: A Cross-Sectional Study" was published in 2022. Journal: Appl Bionics Biomech.

An isokinetic muscle testing protocol was set for the three shoulder movement patterns in the concentric/concentric mode of muscle contraction after system calibration. Angular velocity of 120°/sec was chosen for this study protocol (the recommended testing velocity during the assessment of muscle imbalances) [20]. Moreover, peak torques were normalized to body weight to avoid the effect of weight differences of the participants [21]. Each set consisted of five repetitions as shoulder muscle peak torques were found to be developed during the second or third test repetition in 96% of all cases [22]. Warm up preceded the actual assessment consisted of five minutes of pendulum exercises followed by two sets of dynamic stretching of shoulder flexors, extensors, abductors, adductors, and internal and external rotators, each taking 20 seconds per muscle group [23].

Each participant was positioned in a comfortable sitting position on the Biodex chair with the trunk positioned upright and the hips and knees at approximately 85° flexion. The trunk was supported up to the scapular level by a firm back and stabilized using a combination of pelvic strap and a pair of anterior straps which were stretched diagonally from just above the shoulder level to the opposite pelvic side, crossing each other at the lower part of the sternum. A single strap was applied horizontally across the thigh of the tested side.

Abduction/adduction movement: the participant sat in front of the actuator with trunk upright, hips and knees flexed, elbow extended, and forearm supinated. The mechanical axis of lever arm was aligned with an anatomical point just below the acromion, the dynamometer was tilted 10°, seat oriented at 90 degrees, and seatback tilted 70-85°. The range of movement was set free between the hanging position and 120° shoulder abduction (Figure 2).

The article "Isokinetic Assessment of Shoulder Joint Strength Ratios in Male Recreational Weightlifters: A Cross-Sectional Study" was published in 2022. Journal: Appl Bionics Biomech.

Internal/external rotation movement: the participant sat with trunk upright, hips and knees flexed, and the arm abducted 90° in the scapular plane and supported. The mechanical axis of lever arm aligned to the long axis of the humerus, dynamometer orientated 20° and tilted 10 to 15°, seat orientated 15°, and seatback tilted 55 to 85° according to participant's anthropometric measurement. Limits of the shoulder ROM were set at 30° internal rotation and 90° external rotation so that the shoulder externally rotated throughout a 120° (from 30° internal rotation to 90° external rotation), as shown in Figure 3.

Flexion/extension movement: the participant sat with trunk upright, hips and knees flexed with the axis of lever arm aligned at acromial process in sagittal plane, and seatback tilted 70 to 85°. Limits of the shoulder ROM were set at 60° shoulder extension and 180° shoulder flexion so that the shoulder flexed throughout a 240° (from 60° extension to 180° flexion), as presented in Figure 4.

Afterward, gravity correction was performed for each participant as indicated by the Biodex system 3 manual. Prior to each test, the participant was familiar with the dynamometer by performing three submaximal contractions followed by two maximal contractions at a comfortable speed of 120°/sec, thus preventing negative transfer of learning resulting from performing only submaximal warm ups and then performing maximal tests [24]. Then, two-minute rest was given to each participant before the actual test. A hand-held remote comfort stop was placed in the participant's free hand before the start of any test session. Then, he was instructed to perform one set of five consecutive maximal concentric contractions at 120°/sec angular velocity. All participants received standardized, consistent, and moderate verbal encouragements. Three-minute rest was given between testing positions as it is enough time for adenosine triphosphate repletion [13].

### 2.3. Statistical Analysis

All statistical measures were performed through the Statistical Package for Social Sciences (SPSS) version 20 for windows. It was intended to compare isokinetic concentric shoulder muscle strength values and shoulder muscle agonist/antagonist ratios. Checking normal distribution for each dependent variable, in respect to the independent variable, and detecting outliers were conducted through Shapiro-Wilk normality tests and box plots. To avoid the effect of platykurtic data, *z*-scores for kurtosis were calculated. Data exploration for each set of data revealed that the data of RWL and controls were homogenous and normally distributed. Independent *t*-test was the statistical procedure used to compare the sample means with respect to the dependent variables. The alpha level was set at 0.05.

The article "Isokinetic Assessment of Shoulder Joint Strength Ratios in Male Recreational Weightlifters: A Cross-Sectional Study" was published in 2022. Journal: Appl Bionics Biomech.

## 3. Results

An independent *t*-test, comparing the demographic data between both groups, showed homogeneity of groups in these data except for weight as presented in Table 1. Groups were identified based on participation in recreational weightlifting programs.

Regarding isokinetic concentric-normalized peak torques of assessed shoulder muscles, the mean values of all tested muscle groups were significantly greater in RWL than those of the control group (*p* < 0.05), as shown in Table 2.

Regarding the shoulder joint agonist/antagonist ratios, there was a significant decrease in abductor/adductor and external rotator/internal rotator ratios in RWL compared with the control group (*p* < 0.05). Meanwhile, the statistical difference in the flexor/extensor ratio between both groups was insignificant (*p* > 0.05), as shown in Table 3.

Analysis of exercises: the shoulder adductor muscles were the most targeted muscles during training (94%), followed by shoulder extensors (75%), flexors (73%), internal rotators (71%), and then shoulder abductors (19%), and the external rotator muscles were the least trained muscles (12%). It also revealed that most of muscle groups were exercised for an average of three sets, each set consisted of ten repetitions.

## 4. Discussion

Firstly, the findings of the current study revealed that the tested normalized peak torques of RWL group were significantly higher than those of the control group. The differences in peak torque between both groups were as follows from the highest to the lowest: adductors, extensors, flexors, internal rotators, abductors, and finally external rotators' peak torques. This descending order in the strength values of different shoulder muscle groups matched the specific types of strength exercises performed by the RWL as indicated from the filled exercise sheet by the participants. The strength difference between both groups is attributed to weight training effects. Resistance training results in both muscular and neural adaptations which in turn increase the muscular strength [25]. These adaptations occur as a result of alterations in hormone levels, neuromuscular junction activity, motor unit recruitment, and changes in the contractile proteins in muscle [26].

The findings of the current study are in agreement with those of Barlow et al. [1] who postulated that the selectivity in the training program with special focus on large muscles as pectoralis major, latissimus dorsi, and deltoid muscles with neglection or undertraining of the stabilizers might be the reason for increasing body weight adjusted strength values of shoulder flexors, abductors, and internal and external rotators among body builders as compared with the controls. Moreover, the present study is aligned with the work of Kolber et al. [13] and Kolber and Corrao [14] in terms of the shoulder abductors and internal rotators' strength values. Both studies reported that the increase in these values is referred to overtraining of deltoids and internal rotators among weight training participants as it was indicated by their routine workouts. In addition, Kolber et al. [27] reported that the upper extremity exercise prescription should concentrate on the internal rotation mobility, alleviates training bias, and favors muscles responsible for stabilization, such as the external rotators and lower trapezius.

The article "Isokinetic Assessment of Shoulder Joint Strength Ratios in Male Recreational Weightlifters: A Cross-Sectional Study" was published in 2022. Journal: Appl Bionics Biomech.

Additionally, Kolber and Corrao [14] found a significant increase in the mean external rotator strength value, in the female recreational group compared to the controls. This came in the same context of the present study in spite of the difference in the studied group gender. In the abovementioned study, most of the female participants routinely performed latissimus pull downs towards the body rear. This type of exercise places the shoulder in a position of horizontal abduction combined with external rotation. This shoulder position forces the rotator cuff muscles, along with the external rotators, to work harder to stabilize the head of the humerus [28]. Also, Blache et al. [29] reported that the mechanical work of the rotator cuff muscles, upper trapezius, and anterior deltoid was increased with lifting load and height augmentation.

On contrast to the current study, Kolber et al. [13] found that the difference in shoulder external rotators' strength value between male RWL and controls was not significant. Exercise selection is the key to justifying this disagreement. In the present investigation, participants performed diagonal lateral cable raise and cable external rotation exercises which mainly focus on training of external rotators as prime movers [30]. In addition, they performed reverse butterfly, reverse fly with dumbbells, and shoulder raise lying on the stomach exercises in which external rotators act as stabilizers [30]. With regard to Kolber et al. [13], the only exercise reported by participants that target the external rotators as stabilizers is latissimus pull down to the front [28]. Nonetheless, they did not mention any exercise directly targeting the external rotators.

Another reason for this disagreement may be the difference in testing position. The current study assessed the isokinetic torque of the internal and external rotators, while the shoulder joint is abducted 90°, while Kolber et al. [13] assessed them from a more adducted position. Shoulder adduction changes the length-tension relationship and the line of action of scapulohumeral and axiohumeral musculature putting them in a physiological and biomechanical disadvantage as reported by Davies [31]. Moreover, the training volume should be considered when explaining different strength gains. It was reported that muscle strength gains in response to resistance training are greater with multiple sets per exercise rather than a single set [32]. In the present study, RWL performed external rotator exercises three sets, each set consisted of ten repetitions. On the other hand, exercise parameters were not delineated in Kolber et al.'s [13] study.

The article "Isokinetic Assessment of Shoulder Joint Strength Ratios in Male Recreational Weightlifters: A Cross-Sectional Study" was published in 2022. Journal: Appl Bionics Biomech.

Secondly, the current research revealed a significant decrease in abductor/adductor and external/internal rotator ratios in RWL compared to weightlifters. This can be explained mathematically by the fact that the percent of the increase in adductors and internal rotators' strength values is greater than that of abductor and external rotator strength values, respectively. These results correspond to the fact that the percentage of exercises targeting shoulder adductors and internal rotators is greater than exercises targeting abductors and external rotators, respectively.

Moreover, the recreational weight training group had lower flexor/extensor ratio. However, this decrease was not statistically significant, since the difference between strength mean value between both groups, in flexion and extension, was approximately equal. Also, the percentage of exercises targeting the flexors and extensors was nearly the same. Regarding external rotator/internal rotator ratio, the current result is supported by Kolber et al.'s [13] findings who found that the external rotator/internal rotator ratio decreased significantly in recreational weight training group. They declared that this finding may result from the internal rotators being commonly exercised in recreational weight training as compared to the external rotators, which are usually ignored.

Meanwhile, the current result does not concur with Kolber and Corrao [14] who reported a nonsignificant difference in this ratio between both female groups. It was found that, following resistance training, the absolute strength gain in males is greater than females [33]. Moreover, the self-selected resistance load of women often does not exceed 60% of one-repetition maximum (1 RM) which is suboptimal for increasing the muscle strength [34]. Additionally, the differences in training patterns and exercises, the participants selected in both studies, may account for this disagreement.

The article "Isokinetic Assessment of Shoulder Joint Strength Ratios in Male Recreational Weightlifters: A Cross-Sectional Study" was published in 2022. Journal: Appl Bionics Biomech.

The current study has many clinical implications as it highlights the risk related to adaptations resulting from participation in recreational weight training [35, 36]. Muscle imbalances identified in this study may place RWL at risk of developing many shoulder disorders which in turn affect balance ability and postural stability [37]. It revealed, for example, that shoulder external rotators are the least exercised muscles, even though there is an inverse relationship between the strength of this muscle group and the incidence of shoulder impingement syndrome among RWL [38]. Furthermore, high loads raised overhead in many shoulder weight exercises may predispose RWL to shoulder pain [39]. Additionally, these exercises are performed in either cardinal frontal or sagittal planes at which the rotator cuff and deltoid muscles are at a mechanical disadvantage with increased risks of impingement or subluxation [40]. More specifically, upright row and lateral deltoid raise exercises are performed by 41% and 24% of the participants, and 19% performed both exercises in the present study. These two exercises are strongly related to the development of shoulder impingement syndrome [38].

The major limitation of this study was the fact that isokinetic dynamometer assesses muscle groups, not the torque of specific muscles. As a result, a separate assessment of the mobilizer and stabilizer muscle groups could not be performed. However, it is still utilized as a gold standard in the assessment of muscular performance [41]. Another limitation is that the study was conducted on male RWL due to cultural issues, so the results cannot be generalized on the female population. It is worth noting that this study provides an insight that recreational weight training might alter shoulder biomechanics, whereas future investigation on shoulder kinematics of RWL would be valuable in this respect. Correlational research is also recommended to explore the relationship between antagonistic muscle imbalances in RWL and shoulder injuries.

## 5. Conclusion

Weightlifting training increases the strength of shoulder adductors and internal rotators. Therefore, the restoration of a normal concentric abductor/adductor and external/internal rotator strength ratios may reestablish the muscular balance of shoulder complex and prevent its recurrent injuries.

## Figures and Tables

**Figure 1:** Flowchart of the study procedures.

**Figure 2:** Shoulder abductors and adductors isokinetic testing: (a) initial position and (b) final position.

**Figure 3:** Shoulder external and internal rotators isokinetic testing: (a) initial position and (b) final position.

**Figure 4:** Shoulder flexor and extensor isokinetic testing: (a) initial position and (b) final position.

The article "Isokinetic Assessment of Shoulder Joint Strength Ratios in Male Recreational Weightlifters: A Cross-Sectional Study" was published in 2022. Journal: Appl Bionics Biomech.

**Table 1:** Demographic data of the control and RWL group.

	Control group, *n* = 30	RWL group, *n* = 30	*p* value
Age (years)	20.65 ± 1.87	21.56 ± 3.31	0.331
Weight (kg)	73.39 ± 15.38	84.25 ± 12.88	0.034^∗^
Height (cm)	172.94 ± 8.26	175.34 ± 8.03	0.196
Body mass index (kg/m^2^)	24.90 ± 2.06	26.51 ± 2.13	0.635

Data are presented as mean ± standard deviation. *p* value < 0.05 means significant difference. RWL: recreational weightlifters.

**Table 2:** Data analysis of shoulder muscles normalized concentric peak torques (N.m) at 120°/sec.

	Control group, *n* = 30	RWL group, *n* = 30	*F* value	*p* value
Flexors	60.68 ± 17.15	87.67 ± 10.61	27.322	0.001^∗^
Extensors	56.30 ± 22.21	85.44 ± 17.32	16.433	0.001^∗^
Abductors	52.12 ± 15.19	67.19 ± 12.98	8.762	0.006^∗^
Adductors	38.19 ± 17.68	69.20 ± 22.97	17.886	0.001^∗^
External rotators	32.29 ± 9.94	43.17 ± 5.70	13.729	0.001^∗^
Internal rotators	33.68 ± 17.95	55.86 ± 19.88	10.657	0.003^∗^

Data are presented as mean ± standard deviation. *p* value < 0.05 means significant difference. RWL: recreational weightlifters.

**Table 3:** Data analysis of shoulder muscles agonist/antagonist ratios at 120°/sec.

	Control group, *n* = 30	RWL group, *n* = 30	*F* value	*p* value
Flexors/extensors	1.14 ± 0.26	1.05 ± 0.15	1.326	0.259
Abductors/adductors	1.43 ± 0.44	1.04 ± 0.29	7.804	0.008^∗^
External/internal rotators	1.08 ± 0.34	0.81 ± 0.149	7.847	0.009^∗^

Data are presented as mean ± standard deviation. *p* value < 0.05 means significant difference. RWL: recreational weightlifters.

## Data Availability

The data used to support the findings of this study are available from the corresponding author upon request.
